The article "A Method for Short-Term Prediction of the Metro Station's Individual Energy Consumption Item Based on G-ACO-BP Model" was retracted in 2023. Reasons: suspected computer-generated content; unreliable results or conclusions; concerns about the data; concerns about the results or conclusions.

# A Method for Short-Term Prediction of the Metro Station's Individual Energy Consumption Item Based on G-ACO-BP Model

**DOI:** 10.1155/2021/3474077

**Published:** 2021-10-13

**Authors:** Guorong Sha, Qing Qian

**Affiliations:** ^1^School of Transportation Engineering, Nanjing Vocational University of Industry Technology, Nanjing 210023, China; ^2^Nanjing Chervon Auto Precision Technology Co., Ltd, Nanjing 211106, China

## Abstract

This paper proposes a new method to make short-term predictions for the three kinds of primary energy consumption of power, lighting, and ventilated air conditioning in the metro station. First, the paper extracts the five main factors influencing metro station energy consumption through the kernel principal component analysis (KPCA). Second, improved genetic-ant colony optimization (G-ACO) was fused into the BP neural network to train and optimize the connection weights and thresholds between each BP neural network layer. The paper then builds a G-ACO-BP neural model to make short-term predictions about different energy consumption in the metro station to predict the energy consumed by power, lighting, and ventilated air conditioning. The experimental results showed that the G-ACO-BP neural model could give a more accurate and effective prediction for the main energy consumption in a metro station.

## 1. Introduction

The mileage of domestic urban rail transit has been surging as the construction proceeds in China. As of December 31, 2019, there are 208 completed and officially operated urban rail transit lines in 40 cities in China's mainland with a total mileage of 6736.2 km [1]. The development of urban rail transit increases the power energy consumed dramatically and even becomes the largest power energy consumer of the city. Metro undertakes the lion's share of urban rail transit volume. This vital transport type consumes electricity for vehicle running and station operation. According to the energy consumption statistics of existing metro lines, the vehicle running consumes 50%–60% of the total energy consumption, while 40%–50% of the total energy supports the station operation. The power, lighting, and ventilated air conditioning account for more than 90% of the station energy consumption [2]. Therefore, the major concern in metro operators is how to make and implement effective energy reserve and cost-saving strategies.

Research studies have long focused on the energy consumption prediction of urban rail transit. Prevailing prediction methods include multivariate linear regression method [3], artificial neural network method [4–6], support vector machine [7, 8], genetic algorithm [9], grey theory method [10, 11], and time series method [12].

The article "A Method for Short-Term Prediction of the Metro Station's Individual Energy Consumption Item Based on G-ACO-BP Model" was retracted in 2023. Reasons: suspected computer-generated content; unreliable results or conclusions; concerns about the data; concerns about the results or conclusions.

Most of the above algorithms failed to make accurate predictions. Ant colony optimization (ACO) is a bionic algorithm, which is widely used in overlapping community detection, fault diagnosis, cluster class analysis, power system, and other fields [13, 14]. The ACO offers a practical solution for combinatorial and continuous optimization problems due to its outperforming robustness and optimizing ability. Moreover, the ACO fuses with the G-ACO and other algorithms fast, which has been proved by the successful application to slope displacement prediction [15], social network clustering [16], and medical image boundary extraction [17].

This paper proposed a G-ACO-BP-based prediction model to project the energy consumption item incurred in the metro station, especially short-term energy consumers such as power, lighting, and ventilated air conditioning. The model also offers helpful references to the analysis on the comparison between the existing prediction models and actual energy consumption, exploring the energy-saving potential of the metro station.

## 2. KPCA-Based Selection of Prediction Features of Metro Station's Different Energy Consumption Items

Scholars at home and abroad have researched the influencing factors of metro station energy consumption. Referring to the [18, 19], this paper selected the following 12 inputs, including passenger flow (*x*_1_), 24 hours a day (*x*_2_), holiday (*x*_3_), hourly average temperature (*x*_4_), hourly average relative humidity (*x*_5_), season (*x*_6_), weather characteristic value (*x*_7_), number of station entrances and exits (*x*_8_), number of departure metros (*x*_9_), average illumination (*x*_10_), station size (*x*_11_), and station spacing (*x*_12_), as the input parameters of the G-ACO-BP model. To predict the energy consumption items in metro stations more accurately and effectively, the paper extracts the main prediction features through KPCA. The steps are shown below:

(a) Standardize the 12 influencing factors *x*=[*x*_1_, *x*_2_,…, *x*_12_] according to the following formula:
  (1) $$\begin{array}{c} T_{i}\left(k\right)=\frac{1}{x_{\max}\left(i\right)-x_{\min}\left(i\right)}\left[x_{i}\left(k\right)-x_{\min}\left(i\right)\right], \end{array}$$
where *x*_*i*_(*k*) is the *k*_th_ sampling value of the *i*_th_ influencing factor, *x*_max_(*i*) and *x*_min_(*i*) are the maximum value and minimum value of all sampling points of the *i*_th_ influencing factor, and *T*_*i*_(*k*) represents the standardized target data.
(b) Calculate the kernel matrix *K* according to formula (2) and use the radial basis kernel function to map the original data from the data space to the feature space.
  (2) $$\begin{array}{c} K\left(x_{i},x_{j}\right)=\left(-\frac{\left\|x_{i}-x_{j}\right\|}{2\sigma^{2}}\right). \end{array}$$
(c) Modify the kernel matrix *K* with the centering kernel matrix *K*_*C*_, and the modified formula is
  (3) $$\begin{array}{c} K_{C}=K-l_{N}K-Kl_{N}+l_{N}Kl_{N}, \end{array}$$
where the *K*_*C*_ is the matrix of *N* × *N*, and each element is 1/*N*.
(d) Calculate the eigenvalue of the matrix *K*_*C*_, and its corresponding eigenvectors are *λ*_1_, *λ*_2_,…, *λ*_12_, and its variances are *v*_1_, *v*_2_,…, *v*_12_. The larger the eigenvalue was, the more the useful information it contained. Accordingly, the eigenvectors were adjusted by eigenvalue in descending order.
(e) Orthogonalize and unitize the eigenvectors by adopting the Schmitt orthogonalization method. The eigenvectors obtained were *a*_1_, *a*_2_,…, *a*_12_.
(f) Calculate the cumulative contribution rate *r*_1_, *r*_2_,…, *r*_12_ of the eigenvalue, where the given contribution rate was *p*; if *r*_*t*_ > *p*, the first *t* principal components were selected as the input parameter of the G-ACO-BP model after dimension reduction.

The eigenvalues of the matrix *K*_*C*_ and the cumulative contribution rate of all principal elements are shown in Figure 1. When *r*_*t*_ ≥ 90%, the first five main elements with the largest individual contribution rate in this paper were the passenger flow (*x*_1_), 24 hours a day (*x*_2_), holiday (*x*_3_), hourly average temperature (*x*_4_), and average illumination (*x*_10_).

The article "A Method for Short-Term Prediction of the Metro Station's Individual Energy Consumption Item Based on G-ACO-BP Model" was retracted in 2023. Reasons: suspected computer-generated content; unreliable results or conclusions; concerns about the data; concerns about the results or conclusions.

In the actual operation, the supporting facilities should be built with higher quality, offering more frequent services as the passenger flow in the metro station grows. Such facilities include automatic ticket vending machines, ventilators and air conditioners, and escalators. The working load of those equipment serving in the station should also be enlarged. As a result, the energy consumed by the metro station rises. In the daily 24 hours, the energy consumption at the metro station varies from rush hours to holidays. The temperature at different times in the metro station is related to the energy consumed by as ventilated air conditioning in the metro station. The average illumination in the metro station also directly affects the energy consumed by lighting. According to the theory and the actual situations, we selected five influencing factors, including passenger flow, 24 hours in a day, holiday, hourly average temperature, and average illumination, as the input parameters of the G-ACO-BP model.

## 3. Constructing the G-ACO-BP Model for the Short-Term Prediction of the Metro Station's Different Energy Consumption Items

### 3.1. Constructing the BP Neural Network Model Based on G-ACO

Given the contradiction between the “stagnation phenomenon” and the “blind search” of ACO, this paper selects the genetic-ACO (G-ACO). By combining GA and ACO, the global search capability of the GA-based model would be dramatically improved with the positive feedback convergence mechanism of ACO. First, GA was used to generate pheromone distribution, and then the positive feedback mechanism of ACO was used to find the exact solution. The advantages of the two are complemented and combined to operate.

The article "A Method for Short-Term Prediction of the Metro Station's Individual Energy Consumption Item Based on G-ACO-BP Model" was retracted in 2023. Reasons: suspected computer-generated content; unreliable results or conclusions; concerns about the data; concerns about the results or conclusions.

Since the BP neural network adopted the gradient descent algorithm, the training usually requires longer to achieve convergence and is prone to a local minimum. The G-ACO was fused into the BP neural network to train and optimize the connection weights and thresholds between each layer of the BP neural network. The G-ACO-based BP neural network (G-ACO-BP) model is shown in Figure 2.

In Figure 2, the G-ACO-BP model was an arbitrary neural network with *n*-layer input and *n*-layer output, which contained input, hidden, and output layers. The characteristic of each node was the sigmoid function in which *w* was the weight and *b* was the threshold.

### 3.2. The G-ACO-BP Neural Network Analysis for the Prediction of Individual Energy Consumption Item in the Metro Station

The G-ACO is a global optimization heuristic algorithm used to train and optimize the BP neural network's weights and thresholds. The trained and optimized weights and thresholds underwent error back optimization through BP neural network. The process effectively avoided the defects that could emerge in the BP neural network training, which further optimized the intelligent neural network model [20].

In the G-ACO-BP short-term prediction model of the individual energy consumption item, the G-ACO optimized the BP neural network in the following steps:

(a) Use the genetic algorithm to “digitalize” and encode the energy consumption input samples of the metro station and initialize the population.
(b) Start the cycle: evaluate the fitness of the individual of each chromosome.
(c) Select two individuals from the population as the father and the mother as higher fitness improves the probability of selection.
(d) Choose the chromosomes of the parents for chromosome chiasmata and offspring production.
(e) Mutate the chromosomes of offspring.
(f) Repeat steps (c), (d) and (*e*) until the optimal solution emerges.
(g) Initialize the whole network in ACO. Assume the time was *t* = 0, the number of cycles was *Nc* = 0, *N*_*c*_max__ was the maximum number of cycles, and the information quantity of each element in every set was *τ*_*j*_(*I*_*p*_*i*__)=*C*, and Δ*τ*_*j*_(*I*_*p*_*i*__)=0. Put all ants in the nest.
(h) Activate all ants: for the set *I*_*p*_*i*__, calculate the state transition probability of ants *k*(*k*=1,2,…, *h*) according to the following formula:
  (4) $$\begin{array}{c} \mathrm{Pr}\left(\tau_{j}^{k}\left(I_{p_{i}}\right)\right)=\frac{\tau_{j}^{k}\left(I_{p_{i}}\right)}{\sum_{g=1}^{N}\tau_{g}\left(I_{p_{i}}\right)}. \end{array}$$
(i) Repeat step (viii) until all ant colonies reach the food source.
(j) Suppose *t* ← *t*+*m*; *N*_*c*_ ← *N*_*c*_+1. Use the weights and thresholds selected by the ants to calculate the output value and error of the neural network and record the current optimal solution. After *m* time units, the ants reached the food source from their nest. Update the information quality on each path according to the following formula:
  (5) $$\begin{array}{c} \tau_{j}\left(I_{p_{i}}\right)\left(t+m\right)=\left(1-\rho \right)\tau_{j}\left(I_{p_{i}}\right)\left(t\right)+\Delta \tau_{j}\left(I_{p_{i}}\right),\\ \Delta \tau_{j}\left(I_{p_{i}}\right)=\sum_{k=1}^{h}\Delta \tau_{j}^{k}\left(I_{p_{i}}\right). \end{array}$$
If the *k*_th_ ant chose the element *p*_*j*_(*I*_*p*_*i*__) in this cycle, then
  (6) $$\begin{array}{c} \Delta \tau_{j}^{k}\left(I_{p_{i}}\right)=\frac{Q}{e^{k}}\text{ otherwise }0. \end{array}$$
where *e*^*k*^ is considered as a set of weights and thresholds chosen by the *k*_th_ ant as the output error of BP neural network; it is defined as follows:
  (7) $$\begin{array}{c} e^{k}=\left|O-O_{q}\right|, \end{array}$$
where *O* is the actual output value of the BP neural network and *O*_*q*_ is the expected output value of the BP neural network; the information quantity grew as the error *e*^*k*^ shrunk according to formula (7).
(k) Test the generalization ability of the trained neural network with the verification sample. If the ant colony converged to the optimal path or the number of cycles *N*_*c*_ ≥ *N*_*c*_max__, end the cycle and output the calculation results; otherwise, jump back to step (h) to continue the operation.
(l) The training of the G-ACO-BP neural network: the weights and thresholds under the optimal path were substituted into the normalized learning samples of metro energy consumption by the BP neural network. The optimized weights and thresholds were used for training and testing in the BP neural network.

The above G-ACO-BP neural network training process of the short-term prediction model reflects the energy consumption types in the metro station. According to the model, we summarized the training algorithm into a flowchart in Figure 3.

The article "A Method for Short-Term Prediction of the Metro Station's Individual Energy Consumption Item Based on G-ACO-BP Model" was retracted in 2023. Reasons: suspected computer-generated content; unreliable results or conclusions; concerns about the data; concerns about the results or conclusions.

### 3.3. The Training Process of the G-ACO-BP Network

The flowchart of the G-ACO-BP network when projecting the individual energy consumption item in the metro station is shown in Figure 4.

1. Data acquisition and preprocessing process involves the influencing factors related to individual energy consumption item in the metro station.
2. Analyze the historical data of individual energy consumption in the metro station to establish a database. The database was then normalized with the influencing factors collected. Following these steps, the preprocessed data were divided into training data and test data.
3. Construct the G-ACO-BP network prediction model and optimize the parameter settings, including crossover and mutation probability, information heuristic factor, BP learning rate, and others.
4. Train the G-ACO-BP model with the training data and calculate the error between actual output and target output.
5. Input the test data into the trained G-ACO-BP model for testing and obtain the energy consumption prediction about power, lighting, and ventilated air conditioning.

## 4. The Energy Consumption Prediction of Power, Lighting, and Ventilated Air Conditioning in the Metro Station

The experimental sample data were collected from the hourly monitored energy consumption data of power, lighting, and ventilated air conditioning from March 31, 2019, to April 1, 2020, in a station along Metro Line 3. The 7,320 sets of data for the period from March 31, 2019, to February 1, 2020, were used as training data, while the 1,416 sets of data from February 2, 2020, to April 1, 2020, were used as test data.

### 4.1. Simulation of the G-ACO-BP Model of Energy Consumption Prediction for Power, Lighting, and Ventilated Air Conditioning in the Metro Station

The five influencing factors (passenger flow, 24 hours a day, holiday, hourly average temperature, and average illumination) extracted by KPCA were input with the energy consumption data of power, lighting, and ventilated air conditioning as the input parameters to construct the G-ACO-BP model. The G-ACO-BP model predicts the energy consumption of power, lighting, and ventilated air conditioning from April 2, 2020, to April 8, 2020.

Based on the same historical data, we compared the G-ACO-BP model proposed in this paper with the existing two energy consumption prediction models: the GA-BP model [4] and the ACO model [15]. The prediction values generated by the three models were then compared with the actual values of energy consumption for a given one week. The result is shown in Figures 5–7.

According to Figures 5–7, the predicted value curve of the G-ACO-BP neural network model was more similar to the actual value curve, so the prediction was better than that of the other two models.

The article "A Method for Short-Term Prediction of the Metro Station's Individual Energy Consumption Item Based on G-ACO-BP Model" was retracted in 2023. Reasons: suspected computer-generated content; unreliable results or conclusions; concerns about the data; concerns about the results or conclusions.

### 4.2. Comparison and Analysis of the Energy Consumption Prediction Error of Power, Lighting, and Ventilated Air Conditioning in the Metro Station

The comparisons of the energy consumption prediction error of power, lighting, and ventilated air conditioning of the G-ACO-BP model, the ACO model, and the GA-BP model are shown in Figures 8–10.

As shown in Figures 8–10, the prediction error of the G-ACO-BP model, the ACO model, and the GA-BP model fluctuated around zero. Among them, the fluctuation of the prediction error of the former model was narrower and more stable with higher accuracy and stability during training and learning, thus performing better predictions.

The test adopted the mean absolute error (MAE) and root mean square error (RMSE) as the evaluation benchmarks of the model performance for detailed and specific prediction comparison. By comparing and analyzing the test data, the comparisons of energy consumption prediction error of power, lighting, and ventilated air conditioning of the three models are shown in Table 1. The MAE and RMSE of the G-ACO-BP model were smaller than those of the other two models, which means that the G-ACO-BP model performs better in predicting the individual energy consumption item in the metro station and could produce more reliable predictions.

## 5. Conclusion

This paper establishes a G-ACO-BP short-term prediction model for individual energy consumption items in the metro station. First, we used the KPCA to extract the main factors affecting the metro station's energy consumption. Second, these factors and energy consumption data were set as the input parameters of the G-ACO-BP model. Third, since the BP neural network training required a longer time to converge and was prone to the local minimum, the G-ACO was fused to the BP neural network to train and optimize the connection weights and thresholds between each layer of the BP neural network. Finally, we built a G-ACO-BP short-term prediction model for individual energy consumption items in the metro station to predict consumption value of power, lighting, and ventilated air conditioning. It can be seen from the experimental results in Table 1 that the value of MAE or RMSE is smaller than that of GA-BP and ACO prediction models. The prediction model built in this paper makes more effective and accurate predictions on the short-term itemized energy consumption of metro stations. Research studies on the application of artificial intelligence algorithms in metro station's energy consumption prediction are absent in current literature. Nevertheless, advancing algorithms and large sample data banks will optimize such models to make precise predictions on the metro station's subitem energy consumption in the future. As a result, the engineering practicability of the model will also be enhanced.

The article "A Method for Short-Term Prediction of the Metro Station's Individual Energy Consumption Item Based on G-ACO-BP Model" was retracted in 2023. Reasons: suspected computer-generated content; unreliable results or conclusions; concerns about the data; concerns about the results or conclusions.

## Figures and Tables

**Figure 1:** The eigenvalues of the matrix *K*_*C*_ and the cumulative contribution rate of all principal elements.

**Figure 2:** G-ACO-BP model.

**Figure 3:** Flowchart of the G-ACO-BP neural network training of building's different energy consumption items.

**Figure 4:** The prediction flowchart of the G-ACO-BP network of individual energy consumption item in the metro station.

**Figure 5:** Comparison chart of the power energy consumption prediction.

**Figure 6:** Comparison of the lighting energy consumption prediction.

**Figure 7:** Comparison of the ventilated air conditioning energy consumption prediction.

**Figure 8:** Comparison of the energy consumption prediction error of power.

**Figure 9:** Comparison of the energy consumption prediction error of lighting.

**Figure 10:** Comparison of the energy consumption prediction error of ventilated air conditioning.

**Table 1:** Comparisons of the energy consumption prediction error of power, lighting, and ventilated air conditioning in the three models.

Index	Power			Lighting			Ventilated air conditioning		
	GA-BP	ACO	G-ACO-BP	GA-BP	ACO	G-ACO-BP	GA-BP	ACO	G-ACO-BP
MAE	16.1473	13.3516	6.9419	19.3021	9.7529	4.9311	25.0299	15.1760	9.0303
RMSE	21.9979	16.4869	8.6090	23.9216	11.9649	6.1251	34.5472	22.9845	19.4137

## Data Availability

The data used to support the findings of this study are included within the article.
